This article has been retracted.

# Role of Medical IoT-Based Bone Age Determination in the Diagnosis and Clinical Treatment of Dwarfism Disease Monitoring

**DOI:** 10.1155/2022/7247932

**Published:** 2022-09-30

**Authors:** Shaoxia Wu

**Affiliations:** Linqu People's Hospital, Weifang 262600, Shandong, China

## Abstract

Currently, the prevalence of dwarfism in children in China is about 3%, which is a very large percentage compared with the large population base. With the increase of influencing factors, the prevalence of dwarfism is on the increase. However, there is a lack of awareness of dwarfism among parents and a lack of in-depth analysis of the causes of dwarfism and a low level of treatment among doctors. Early expert system knowledge base relies on manual editing, which is a traditional, semi-intelligent auxiliary diagnostic system, and is unable to perform disease diagnosis and clinical treatment monitoring well. Many studies have turned to the combination of IoT for bone age determination and its role in the diagnosis and monitoring of clinical treatment of dwarfism. In this study, 15 children with short stature who underwent health checkups at a hospital were enrolled in the study, and a G-P spectrum method was used to determine the bone age of all the enrolled subjects, and the results obtained in the process of bone age determination were systematically analyzed. The results showed that the bone age measurement technique has sufficient reference value for evaluating the quality and diagnosing diseases, and the research and development of this technique is of great significance for the development of modern clinical medicine.

## 1. Introduction

Dwarfism is regulated by endocrine hormones, which prevent children from growing taller normally, and is also influenced by factors such as growth environment and parental height. The incidence of dwarfism is on the rise as the number of influencing factors increases [1]. According to surveys, 90% of children with short stature have varying degrees of low self-esteem, depression, introversion, and other psychological or behavioral disorders, which may affect their schooling, employment, and marriage. Patients with short stature have a variety of negative personalities and are prone to fatigue such as weakness, reduced activity, poor concentration, memory loss, and inefficient learning [2], and fatigue can induce more negative emotions [3]. Short stature not only affects the patients themselves but also the society. It can cause serious psychological problems, work, and life obstacles for patients. The society also needs to pay attention to the inconvenience of work and life of short stature patients, which increases the cost to the society. Short stature is an unfavorable factor that endangers people's physical and mental health and affects social stability and harmony, so dwarfism is getting more and more attention from parents, teachers, and society. We must do early screening, diagnosis, and treatment for children with the disease, which will have a very important significance.

The causes of dwarfism are very complex, which makes it more difficult for doctors to diagnose as well as treat the condition. Even for endocrinologists, misdiagnosis often occurs. In remote areas where medical care is not well developed, missed diagnosis, underdiagnosis, and misdiagnosis are more common [4]. With the increasing concern about children's height, the increasing awareness of the dangers of dwarfism, and the increasing understanding of the mental health of patients with dwarfism, more and more researchers have joined the scientific research on the diagnosis and treatment of the causes of dwarfism [5].

With the development of artificial intelligence and the accumulation of medical data, intelligent assisted diagnosis has been widely used in the medical field. The early intelligent assisted diagnosis was mainly in the form of expert systems. Expert systems are a branch in the field of artificial intelligence [6]. A large number of researchers in the field of medicine have done a lot of work and made progress in the area of expert systems. The most famous of them is Liu et al. of Stanford University who developed the medical diagnostic system MYCIN for blood infections in 1971, which deduces the infecting bacteria and gives a treatment plan based on the patient's symptoms, medical history, and blood test results [7, 8]. MYCIN is a typical example of the success of expert systems. Miller and other scholars from the University of Pittsburgh, USA, developed Internist-I, a computer-aided diagnostic system for internal medicine, in the 1980s [9]. Alikeles et al. in Turkey developed an expert system for breast cancer diagnosis using a fuzzy neural network approach. In China, in 1978, Professor Guan Youbo and his team from Beijing College of Traditional Chinese Medicine jointly summarized Professor Guan's experience in the treatment of liver diseases and developed the liver disease diagnosis and treatment system, which was the first expert system in China. Expert systems in the medical field have also emerged in recent years, including kidney expert systems, diabetes expert systems, and other expert systems for various diseases.

The traditional expert system for disease diagnosis has obvious shortcomings, and it has several shortcomings.

1. The “bottleneck” problem of knowledge acquisition: the empirical knowledge of each expert is subjective, and it is also required that these medical experts have certain computer knowledge; otherwise, it is difficult to describe the knowledge by rules, which is not conducive to the establishment of knowledge base.
2. Poor adaptability of the system: the establishment of the knowledge base is all dependent on manual editing, which cannot learn independently and has no ability to learn knowledge from historical experience.

## 2. Related Work

The causes of dwarfism are complex, and there are different treatments for different causes. The main etiologies are as follows:

1. Growth hormone deficiency: the etiology can be divided into primary and secondary. Primary growth hormone deficiency can be caused by genetic inheritance and is classified as I (AR), II (AD), and III (X-linked) according to the mode of inheritance. Primary growth hormone deficiency can be caused by pituitary hypoplasia or hypopituitarism, or the hypothalamus and pituitary gland do not have any obvious foci, but the growth hormone secretion function is insufficient. It can occur at any stage of the child's growth.
2. Idiopathic dwarfism: idiopathic dwarfism [10] is a temporarily unspecified cause of dwarfism and is one of the most common types of dwarfism.
3. This type of dwarfism is usually due to the mother's own disease at the time of pregnancy, such as maternal gestational hypertension and maternal smoking and drug use, which can cause intrauterine growth retardation. This type of fetus is usually born with a long body and is characterized by low weight, which must be diagnosed and treated early to avoid serious effects on its lifelong height [11].
4. Familial dwarfism: familial dwarfism is caused by genetic predisposition to dwarfism. Usually, both parents of the affected child are short, or one of the parents is normal and the other is short, or there is a close relative with short stature [12].
5. Turner syndrome: it is a common disorder with abnormal number or structure of sex chromosomes. Typical children with Turner have characteristic physical and phenotypic abnormalities, such as wide eye spacing, ptosis, entropion, short neck, multiple nevi or milk coffee spots, elbow ectropion, low hairline, high palatal arch, and shield chest.
6. Chondrodysplasia: osteogenesis imperfecta is due to disorders of connective tissue. This means that collagen formation is impaired, leading to congenital genetic disorders. Chondrodysplasia is a congenital dysplasia due to defective endochondral ossification, which mainly affects long bones and is clinically manifested as a specific type of dwarf-short-limbed dwarf.

As one of the important components of “Smart Earth,” medical IoT refers to the application of IoT-related technologies to share and connect medical information and establish a unified, efficient, real time, and interoperable system for disease research, prevention, diagnosis, and treatment, so that patients or healthy people can receive timely, convenient, and equitable medical and health services in real time without the limitation of space and time [13]. This will enable patients or healthy people to receive timely, convenient, and equitable medical and health services in real time without space and time constraints [14]. Medical IoT system is based on the existing public health information platform and uses IoT-related technologies to form an information network integrating command, emergency response, and management supervision by integrating information from public health systems at all levels. A high degree of collaboration between patients and medical equipment, hospitals, and public health organizations is achieved, and the overall informatization of the medical industry is gradually realized [15].

China's medical IoT system started in 2004, which is a late start compared with developed countries, and its development history is shown in Figure 1. At this stage, the construction of medical IOT system in China is gradually transitioning from the primary stage of hospital information based on revenue and expenditure management to the advanced stage based on clinical information [16, 17], and steadily realized the transformation from “cost-centered” to “patient-centered” [18]. The shift from “cost-centered” to “patient-centered” has been steadily achieved [19]. At present, most hospitals have already started the construction of medical IoT systems, most of which are based on hospital information system (HIS), and the application of HIS is basically mature and gradually expanding. Clinical information system (CIS), medical image storage and transmission system, radiology information system, and other systems are gradually matured and promoted, but the integration is difficult and the development is slow at present. Compared with foreign countries, the domestic medical IOT system still has a large gap; according to the data disclosed at the 2020 Chinese Hospital Information Network Conference, in 2019, the average application level of electronic medical records in China's tertiary hospitals is 3.11, and the average application level of secondary hospitals is 1.59, and as of 2019, only 85 medical institutions in China have passed level 5 and above, and the average score of national hospital wisdom service rating is only 0.33, while the percentage of hospitals in the United States that have passed HMISS level 5 and above has been as high as 70% in 2017 [20]. Moreover, due to the low overall scale of medical IoT investment in China, the system interconnection between different suppliers is difficult, the degree and efficiency of information integration are low, the data entry time is long, and the platform construction is repeated [21].

With the gradual promotion of medical IoT in China, the data output of hospitals is growing geometrically, which has put forward higher requirements for medical data storage. The management of medical data through the cloud has the feature of on-demand distribution, and cloud technology has been able to virtualize storage resources, servers, etc., providing a solution for the growing demand of medical data storage and management. At the same time, due to the unbalanced and insufficient regional development of the domestic healthcare industry, and compared with the proportion of information construction investment in the total annual budget of hospitals in developed countries, most hospitals in China have a considerable gap and slow growth in investment [22]. Therefore, the medical IoT system will gradually develop regionally, with one or more tertiary hospitals in the region as the center, and connect in a radial way. Therefore, the medical IoT system will gradually develop regionally, with one or more tertiary hospitals in the region as the center, and connect all hospitals and public health institutions in the region in a radial way, thus realizing the sinking of high-quality medical resources [23]. In addition, the development of medical IOT system will provide an important way and means to combat and prevent public health emergencies in the future, and at the same time, it will be a significant help to improve the level and quality of medical services in backward regions.

## 3. Methodology

In this paper, the medical IoT system based on IoT technology can be divided into 4 layers of architecture, see Figure 2.

At present, the clinical definition of dwarfism in China is based on the standard deviation method and the height percentile method, or if his or her height is less than the 3rd percentile of the height of children in that population.

It is important to note that some children below 2 SD may still be normal. In other cases, children with normal stature may have a sudden growth arrest and should be diagnosed as soon as possible, even though their height has not fallen below the mean height of -2 SD of normal children of the same sex and age.

Before diagnosing the cause, we first diagnose the child as a dwarf according to the definition of dwarfism and then diagnose the cause according to the indicators obtained from history taking, physical examination, laboratory tests, and imaging tests. The diagnostic approach is divided into clinical and laboratory approaches. The clinical approach is based on physical examination, and the laboratory approach is based on laboratory tests and imaging tests.

The clinical concept is based on the physical examination indicators, such as growth rate, uniformity of body shape, obesity or thinness, and the presence of skeletal deformities, to broadly classify the cause of dwarfism. The clinical idea of the diagnosis is shown in Figure 3.

When physical examination does not provide sufficient clues, laboratory tests and imaging should be performed to find the cause of relatively insidious growth arrest. Laboratory tests are performed to detect thyroid function, chromosomes, growth hormone, bone age, sex hormones, and other indicators to classify the specific causes of dwarfism in detail. The laboratory concept of the diagnosis is shown in Figure 4.

### 3.1. History Taking

Adult lifetime height is often related to genetics (e.g., race, family, early or late sexual maturity, good or bad nutritional status), maternal conditions (e.g., maternal nutrition, mood, disease status, presence of obstetric malformations, exposure to drugs, radiation, alcohol, and tobacco), personal nutrition, presence of disease, presence of hormonal deficiencies, and living and growing environment, so history taking should pay attention to the above mentioned aspects.

Medical history taking includes personal history, maternal and maternal history, past history, and family history.

Personal history includes birth history to understand the fetal growth (gestational age, delivery method, birthweight, birth length, whether asphyxia, etc.) and to inform the doctor of the onset of puberty (early or late) and the age of onset of growth retardation, etc., so that the doctor can grasp the full picture of the child's growth and development stages.

Maternal pregnancy history: the mother's pregnancy is a life-growing process, so her pregnancy history may affect the later growth and development of the fetus. It is necessary to know whether the mother has a history of miscarriage, the number of fetuses, the number of births, whether she has a history of taking medication during pregnancy, whether she has smoked and taken drugs during pregnancy, and whether she has other symptoms such as high blood pressure.

Past history: we need to know whether the child has a history of traumatic brain injury, intracranial infection, tumor, surgery, nutrition, obesity, psychological injury or IQ problems, etc.

### 3.2. Physical Examination

The physical examination includes checking the height and weight of the child, observing the child's facial appearance (to see whether there is a large head, prominent forehead, wide eye spacing, canthus, nevus, cataract, etc.), checking whether the figure is even, whether the body shape is symmetrical, whether there are deformities in the limbs, and checking the development of the child's secondary sex characteristics. It also includes physiological function tests, such as pulmonary function indicators, cardiovascular function indicators, and muscle strength indicators. Among them, height and weight checks are particularly important.

After data preprocessing, Chinese word separation of electronic medical records, and construction of custom dictionaries, the obtained feature words are not directly available as features for model classification. Which words can be used as feature attributes of dwarfism to train the model is the focus of the next research. In this paper, after the subword classification of electronic medical records, TF-IDF statistics is performed. However, it happens that some words that are less relevant to the diagnosis of dwarfism have high TF-IDF values. There are no pasturing area, mining area, high fluorine area, and low iodine area life history and no history of drug use. The words after these subscripts tend to appear more frequently in this document and less frequently in other documents. However, they are not significant for the diagnosis of the etiology of dwarfism, so they can be excluded from the feature candidates.

The remaining words were used as feature candidates after removing some words with high frequency but useless words by word separation. The best features of this research were obtained by combining data-driven and knowledge-driven (Table 1).

After determining the attributes, from the original data, the attribute values corresponding to each attribute in each data entry are extracted. Since some of the descriptions of the bone age item in the electronic medical record are numerical, it is necessary to compare the bone age value with the age value to determine whether it is backward or normal when extracting the attribute values. Since not every data entry will have karyotype and CT/MRI test values, the missing values need to be filled in. Because these two items are nonessential tests, when they are vacant, the default is that both chromosome and CT/MRI values are normal. After a series of processing such as electronic medical record parsing and Chinese word separation, the semistructured electronic medical record is transformed into structured data.

The next step is to numerically process the attribute values of the existing structured data. For the gender attribute, the attribute value of male is marked as 0 and the value of female is marked as 1; the bone age is marked as 0 and the backwardness is marked as 1; the uniform body is marked as 0 and the deformity is marked as 1; and the normal puberty is marked as 0 and the early puberty is marked as 1. The final processing results are shown in Table 2.

## 4. Case Study

In order to determine more clearly and visually whether a child suffers from dwarfism, this study was summarized for the standard height of children, as shown in Figures 5 and 6.

Specific clinical ideas are shown in Figure 7.

If a patient with short stature is encountered in the clinic, normal children of the same region, sex and age should be compared with those whose height is -3 SD.

1. For those below -3 SD in height, they should be screened immediately for routine etiology and their pituitary function should be examined.
2. For height between 2 and 3 SD of normal child height, screening tests for conventional etiology should be performed and, if no abnormality is found, the growth rate should also be observed for at least 6 months.
3. For children whose height is between 0 and 2 SD of normal height, the growth rate should be observed for at least 6 months before deciding whether to examine them for the cause of the disease.
4. When the growth rate is below the 3rd percentile of normal children, etiological examination should be performed regardless of whether their height is normal or not.

In this study, 103 children who visited the pediatric department of a city people's hospital for dwarfism were selected for observation and analysis.

History taking is maternal pregnancy and birth, history of asphyxia, feeding history, growth and development, and disease history.

Physical examination is measure height, body mass, and observe the trunk, limbs, and face of the child for any abnormalities.

Laboratory tests: bone age testing was performed using left-handed orthopantomogram and G-P spectrum method bone age assessment using Jinsai Short Height Assisted Diagnosis and Treatment Monitoring software. Spine, thorax, pelvis, and extremities were performed for suspected abnormal skeletal development to clarify the etiology. For chromosomal examination mainly for girls, some boys with physical abnormalities, and girls, uterus, and ovaries were examined, and children with sexual development were evaluated with GnRH stimulation test if necessary.

ANOVA was taken to further analyze the mean values of children with different etiologies of bone age backwardness. Etiological analysis: among 103 children, the diseases causing dwarfism were idiopathic dwarfism (ISS) 45.7%, growth hormone deficiency (GHD) 22.2%, less than gestational age (SAG) 9.2%, somatic delayed puberty 5.9%, hypothyroidism 3.3%, Turner syndrome 3.3%, polypituitary hormone deficiency 2.9%, precocious puberty 2.3%, and chondrodysplasia 1.3%, as in Table 3.

The bone age development of children with different etiologies of dwarfism: statistical statistics on the bone age lag between groups with different etiologies showed statistically significant differences, as shown in Table 4.

Endocrine disorders are the most common causes of childhood dwarfism. The proportion of ISS and GHD in this study was significantly higher than in all groups. The higher proportion of ISS was related to the fact that a city is a southern inland region with a predominantly agricultural population and the low basal height of the parents of the children. The analysis of the reason for the higher proportion of GHD may be related to the fact that some children with non-GHD dwarfism were excluded from GH motor stimulation tests before inclusion.

This study shows that endocrine disorders are the main cause of childhood dwarfism, and one of the common disorders is GHD. Inquiries into their medical history reveal that about 20% of the children have an abnormal birth history, including a history of fetal malposition or birth asphyxia, which shows that GHD has an important relationship with a variety of diseases in the perinatal period, in which the neurological (pituitary cells) damage due to HIE is the most significant. Therefore, avoiding difficult birth asphyxia is important to reduce the occurrence of GHD. ISS accounted for 15.7% of children with dwarfism in this study. There are individual differences in the treatment effect of ISS using GH; therefore, further genetic testing is needed in clarifying the cause. Except for GHD and ISS, the incidence of other diseases is relatively low, including 28 cases (9.1%) of less than gestational age (SAG). Although most SGAs may have a substantial increase in growth after 2 years of life, nearly 1/4 of SGAs are still born with growth retardation and fail to achieve catch-up growth, thus leading to short stature in adulthood. Based on this current situation, it is critical to enhance maternal health care to minimize the causative factors causing SCA and to strengthen the monitoring of growth after birth of SGA. Among them, there were 10 cases (3.2%) of hypothyroidism. Although in China, screening for neonatal diseases has been carried out for decades, there are still a few children with hypothyroidism who are underdiagnosed, so it is necessary to perform routine thyroid function tests in children with short stature. Among them, 10 cases (2.9%) of Turner syndrome are with diverse karyotypic manifestations but mostly atypical clinical manifestations; for girls with short stature, special attention was paid to the presence of TS signs and routine chromosome examination.

Analysis of age characteristics and bone age development in children with different causes of dwarfism: we analyzed the characteristics of bone age in children with different causes of dwarfism, and the results showed that the bone age of children with the same cause of dwarfism was less than the actual age in different degrees. Among them, growth hormone deficiency, hypothyroidism, and Turner syndrome had the most significant bone age lag, while familial dwarfism and children younger than fetal age had less bone age lag. There are three main factors that have a significant impact on the bone age of children, namely, thyroid hormone, sex hormone, and growth hormone. Once the child has insufficient growth hormone secretion or hypothyroidism, the bone age will be backward. Thus, when a child with short stature has no delay in bone age, it should be considered that the growth disorder is not related to insufficient growth hormone or hypothyroidism. In addition, bone age is also commonly used clinically for the assessment of clinical medication and treatment effects.

## 5. Conclusion

At present, with the attention of parents, teachers, and society to the problem of childhood dwarfism, more and more endocrinologists begin to pay attention to the childhood dwarfism. However, children's growth is affected by genetic factors, nutritional factors, disease factors, and neuroendocrine factors. The analysis of the pathogenesis of dwarfism varies from region to region. Therefore, this paper discusses the causes of dwarfing and aims to develop a model and system of artificial diagnosis of dwarfism based on the combination of medical materials, help doctors effectively control auxiliary diagnosis and clinical treatment, improve the curative effect of experts, and realize the early diagnosis and treatment of dwarfism, which is very important to improve the growth of short children and the quality of life of local residents. At the same time, it is also necessary to strengthen publicity and education for parents to make them pay attention to the growth and development of children, and ensure early detection and timely treatment, so as not to ignore the best treatment opportunities.

## Figures and Tables

**Figure 1:** Development history of medical IoT system in China.

**Figure 2:** Overall framework of medical IoT system based on IoT technology.

**Figure 3:** Clinical thought diagram for diagnosis.

**Figure 4:** Laboratory thought diagram for diagnosis.

**Figure 5:** Change curve of height and weight of male children.

**Figure 6:** Change curve of height and weight of girls in China in 2005.

**Figure 7:** Diagnostic process of dwarfism.

**Table 1:** Description of attributes.

Serial number	Property name	Description
1	Sex	Depending on the gender of the child, the doctor will perform different tests. Gender is divided into male and female
2	Growth rate	The number of centimeters of growth per year is used to determine whether the child is growing slowly or normally. In general, children between the ages of 1 and 18 grow 1–8 cm per year.
3	Body mass	We can determine whether the growth is uniform or deformed by looking at the size of the child.
4	Bone age	Bone age is examined and compared with the true age. The values are normal bone age and lagging bone age.
5	Father's height	To determine whether the father is short by checking the father's height.
6	Mother's height	The height of the mother was examined to determine whether the mother was short.
7	Family history	To determine whether the height of close relatives in the family is hereditary or not. The values are yes and no.
8	Maternal smoking during pregnancy	To check whether the mother smoked during pregnancy and the age of smoking. The range of values is 0–30.
9	Maternal hypertension during pregnancy	To check whether the mother had high blood pressure during pregnancy. The values were yes and no.
10	Maternal pregnancy hypertension	To check whether the mother has hyperemesis during pregnancy. The values were yes and no.
11	Adolescence	To find out the time of puberty. Values are normal, early.
12	Thyroid function	The values of FT3 and FT4 in laboratory tests are normal and abnormal. The values are normal and abnormal.
13	Chromosome karyotype	In special cases, the karyotype of the chromosome is examined. The values are normal and variable.
14	CT/MRI	The size of the pituitary gland and the presence of occupational lesions are observed. The values are normal and abnormal.

**Table 2:** Partial data after numerical attribute value.

Sex	Bone age	Body mass	Growth rate	Adolescence	Maternal pregnancy symptoms	…	LH/PSH	GH	Thyroid function	IGF-1	Chromosomes	CT/MRI
0	1	0	0	0	0	…	0.45	0.88	0	1	0	0
0	0	0	3.4	0	1	…	0.31	4.33	0	0	0	0
0	1	0	4.3	0	0	…	0.88	1.22	1	0	0	1
1	1	1	2	0	1	…	0.24	3.67	0	1	1	0
…	…	…	…	…	…	…	…	…	…	…	…	…
0	1	0	4	1	1	…	1.76	12.67	1	0	0	0
1	0	0	3.6	0	1	…	0.53	4.36	0	1	0	0
1	1	0	4	0	0	…	0.54	10.08	0	1	0	0
1	0	0	6	1	1	…	1.24	3.69	0	1	0	0
1	1	1	4	0	0	…	10.20	10.22	0	0	1	0
1	1	0	1	0	0	…	0.90	0.88	0	1	0	0

**Table 3:** Distribution of the number of cases and number of cases at different ages for the etiology of 103 children with dwarfism.

Etiology	Number of cases [*n*%]	＜6 years old	Undeveloped over 6 years old	Developed over 6 years old
Complete GHD	3 (4.3)	1	8	5
Partial GHD	5 (18.1)	8	38	9
ISS	39 (45.5)	36	77	26
Familial dwarfism	13 (3.7)	3	4	5
SGA	9 (9.0)	7	19	3
Thyroid function	9 (3.4)	1	7	1
Somatic delayed puberty	7 (5.8)	0	5	11
Turner syndrome	11 (3.2)	1	4	1
Precocious puberty	7 (2.4)	0	10	7
MPHD	9	1	0	0
Chondrodysplasia	4	4	8	0

**Table 4:** Comparison between age and bone age development of children with different etiologies of dwarfism ($\bar{x}\pm s$).

Etiology	Number of cases	Age	Bone age	Age difference
Complete GHD	3	10.85 ± 3.11	8.39 ± 2.81	1.463 ± 0.68
Partial GHD	4	9.3 ± 2.93	6.97 ± 2.72	2.263 ± 0.56
ISS	39	8.31 ± 2.95	7.35 ± 2.87	0.955 ± 0.75
Familial dwarfism	13	9.92 ± 3.52	9.29 ± 3.57	0.584 ± 0.49
SGA	9	7.62 ± 2.69	6.55 ± 2.47	1.06 ± 0.53
Thyroid function	9	10.51 ± 1.99	6.13 ± 2.11	4.31 ± 1.79
Somatic delayed puberty	7	14.88 ± 0.75	10.64 ± 0.79	4.15 ± 0.69
Turner syndrome	11	9.35 ± 2.82	7.25 ± 2.33	4.19 ± 0.62
MPHD	9	9.32 ± 2.89	7.25 ± 2.53	2.03 ± 0.81
*F*		12.506	5.686	86.682
*P*		<0.001	<0.001	<0.001

## Data Availability

No data were used to support this study.
